# Effects of Sevoflurane on Apoptosis of Myocardial Cells in IRI Rats

**DOI:** 10.1155/2021/3347949

**Published:** 2021-12-31

**Authors:** Shikun Zhang, Xiaoyan Du, Kun Zhang, Haiyan Wang

**Affiliations:** ^1^Department of Cardiovascular Disease, Gaomi People's Hospital, 77 Gaomi Zhenfu Street, Weifang, 261500 Shandong, China; ^2^Department of Ophthalmology, Gaomi People's Hospital, 77 Gaomi Zhenfu Street, Weifang, 261500 Shandong, China; ^3^Department of Geriatrics, Gaomi People's Hospital, 77 Gaomi Zhenfu Street, Weifang, 261500 Shandong, China

## Abstract

**Background:**

Cardiomyocyte apoptosis functions essentially in ischemia/reperfusion- (I/R-) induced myocardial injury. It is suggested that autophagy is widely implicated in the regulation of cell survival and death. Sevoflurane, as a largely used inhalational general anesthetic, has been shown to have a protective effect on cardiomyocytes. However, it was yet elusive on the underlying mechanisms.

**Aim:**

The objective of this study is to investigate the association of sevoflurane-mediated cardioprotective effects with autophagy regulation.

**Methods:**

An in vitro hypoxia model was established in primary cardiomyocytes from fresh myocardial tissue of the rats. The apoptosis rate of myocardial cells treated with hypoxia and treated with sevoflurane was measured. Western blot and immunocytochemical assay were used to measure the protein expression. The cell proliferation rate and cell apoptosis were measured using the MTT assay and flow cytometry, respectively.

**Results:**

The expression of apoptotic proteins including B cell lymphoma-2 (Bcl-2), CCAAT/enhancer-binding protein homologous protein (CHOP), glucose-regulated protein 78 (GRP78), and Bcl-2-associated X protein (BAX) in myocardium treated with sevoflurane was significantly lower than that in myocardium treated with hypoxia. The expression of adhesion proteins such as intercellular adhesion molecule-1 (ICAM-1), vascular cell adhesion molecule-1 (VCAM-1), and E-selectin in myocardium treated with sevoflurane was higher than that in myocardium treated with hypoxia, suggesting better connectivity of the myocardium.

**Conclusion:**

Sevoflurane treatment reduced the apoptosis of myocardial cells after hypoxia treatment.

## 1. Introduction

General anesthesia is a reversible state induced by drugs [1]. Under the condition of maintaining physiological stability, patients will have a reversible state such as coma, forgetfulness, antisyncope, and immobility [2]. Since the first public display of diethyl ether as a general anesthetic at Massachusetts General Hospital (MGH) in 1846, the practice of anesthesiology has revolutionized surgery and spurred the advance of modern medicine [3]. Today, more than 170 years later, the administration of diethyl ether derivatives remains the basis of anesthesiology [4]. Fluoromethyl hexafluoroisopropyl ether, also known as sevoflurane, is a derivative of diethyl ether, which is widely used in current clinical practice [5].

The change of diet and the improvement of living standard make the incidence of cardiovascular disease in China rise rapidly [6]. At present, the main treatment method is to restore normal blood supply to the heart by recanalization of blocked coronary arteries by surgical operation or intervention. Cardiac surgery is more susceptible to external factors than surgery on other solid organs, so anesthesia is more carefully used [7]. Improper use or concentration of anesthetic drugs can cause patients with arrhythmia, tachycardia, bradycardia and other symptoms, or even death [8].

Sevoflurane, as a new sort of inhalation anesthetic, produces excellent anesthesia quality and is commonly employed in cardiac surgeries since it exerts more fast and smooth recovery than other inhaled anesthesia. It was demonstrated that the application of sevoflurane at the onset of reperfusion (sevoflurane postconditioning) was a protective stimulus to decrease ischemia/reperfusion (I/R) injury in patients undergoing coronary bypass surgery [9]. Studies have found that sevoflurane can not only improve the myocardial contractility but also reduce the myocardial infarction area, which has a protective effect on the myocardium [9, 10]. Sevoflurane pretreatment of isolated rat right ventricular muscle can effectively promote the recovery of myocardial contractility after reperfusion. Studies have shown that sevoflurane pretreatment and posttreatment can both reduce the area of heart infarction, but posttreatment is more widely used than sevoflurane preconditioning in clinical therapy [9]. Additionally, *in vivo* studies and clinical observations have shown that sevoflurane can increase left ventricular pressure (LVDP) and reduce left ventricular end-diastolic pressure (LV-EDP) [11].

Therefore, in this study, we aimed to investigate the effects of sevoflurane treatment in rat-derived primary cardiomyocytes. We demonstrated the protective effect of sevoflurane on hypoxic cardiomyocytes. And this protective effect was demonstrated by reducing the expression of apoptotic proteins in myocardial cells.

## 2. Methods

### 2.1. Primary Cell Culture

The fresh myocardial tissue of the rats was cut into 1–2 mm^3^ heart fragments in phosphate-buffered saline (PBS) containing 0.1% trypsin and 0.1% collagenase. After the digestion of tissues 3-4 times, 5 minutes each time, the digested cells from the tissues were collected and centrifuged in DMEM containing 10% FBS. Finally, the cells were cultured in DMEM containing 10% FBS. The cell suspensions were mixed and plated at a cell culture flask in 37°C in a 5% CO_2_ incubator for 30 min cultivation. The cells were then cultured in 6-well and 96-well plates and kept at 37°C and 5% CO_2_. On the first 2 days, 100 mM 5-bromo-29-deoxyuridine (BrdU; BioVision, USA) inhibits nonmyocyte proliferation. The cells were cultured for 3 days.

### 2.2. Hypoxia Treatment and Experimental Grouping

For hypoxia treatment, oxygen-control incubator (Thermo Fisher Scientific Inc., Waltham, MA) was used. Cardiomyocytes were randomly divided into three groups. To study the protective effect of sevoflurane against hypoxia in cardiomyocytes, cells cultured under normal oxygen conditions (normal control) were set up. Cells were cultured in an anaerobic chamber with 2% CO_2_ and 95% N_2_ for 24 h (hypoxia group). For anesthetic agent treatment, cells pretreated with 1.8 mg/mL sevoflurane were incubated in an anesthesia induction chamber immediately after hypoxia treatment at 37°C, 2% O_2_ for 12 h (hypoxia+sevoflurane group).

### 2.3. Cell Viability

The effect of sevoflurane on cell proliferation was determined using the MTT method.

Briefly, the cells were treated as described above and were placed in a 96-well plate and cultured overnight in DMEM and 10% FBS containing 0.5 mg/mL of MTT (Biotech, Shanghai, China). An automated microplate reader was used to measure the absorbance at 490 nm (Molecular Devices, Sunnyvale, CA).

### 2.4. Flow Cytometry Assay

After different treatments, the cells were plated in six-well plates. The medium was replaced with cold 75% ethanol to fix the cells at 4°C overnight. Then, 10 *μ*L of Annexin V-fluorescein isothiocyanate (FITC) binding buffer (Sigma-Aldrich, USA) and 5 *μ*L of propidium iodide (PI) (Sigma-Aldrich, USA) were added to each well to incubate cells for 20 min in the dark. The apoptosis rate of each well was detected by using a FACScan flow cytometer (Beckman-Coulter, California, USA).

### 2.5. Western Blot

Western blot was performed to detect then expression levels of B cell lymphoma-2 (Bcl-2), CCAAT/enhancer-binding protein homologous protein (CHOP), glucose-regulated protein 78 (GRP78), Bcl-2-associated X protein (BAX), intercellular adhesion molecule-1 (ICAM-1), vascular cell adhesion molecule-1 (VCAM-1), and E-selectin in the heart cells from control, hypoxia, and sevoflurane groups. Cells were homogenized and protein isolated using the RIPA lysis buffer system (Thermo Fisher, Massachusetts, USA). Protein concentrations were quantified using the BCA protein assay (Beyotime, Shanghai, China), and all samples were loaded with equal protein onto 10% polyacrylamide gel with 0.1% sodium dodecyl sulfate (SDS). Proteins were then separated by electrophoresis and transferred onto nitrocellulose membranes. Nonspecific binding sites were blocked with Tris-buffered saline solution (TBS) containing 5% dry milk. The membranes were incubated with primary antibodies against ICAM (ab171123, Abcam; 1 : 500), E-selectin (ab18981, Abcam; 1 : 1000), VCAM (ab134047, Abcam; 1: 500), Bcl-2 (ab32124, Abcam; 1 : 500), BAX (ab32503, Abcam; 1 : 500), GRP78 (ab21685, Abcam; 1 : 500), and *β*-actin (ab8226, Abcam; 1 : 1000). After the membranes were cleaned, protein blots were detected by enhanced chemiluminescence (ECL) (Beyotime). The intensity of the identified bands was detected by densitometry software (Quantity One software; Bio-Rad, Hercules, CA, USA).

### 2.6. Statistical Analysis

The representative data were expressed as the mean ± standard deviation (SD) from three independent experiments. SPSS version 19.0 software (IBM Corp., Armonk, NY, USA) was employed for statistical analysis. Data among multiple groups were compared with one-way analysis of variance (ANOVA), and data between two groups were compared by Student's *t*-test. A *P* value < 0.05 was considered to be statistically significant.

## 3. Results

Flow cytometry was used to analyze the cell death of myocardial cells in three groups (control group, hypoxia group, and hypoxia+sevoflurane group). Compared with the control group, 12-hour hypoxia treatment resulted in a large number of myocardial cell apoptosis (Figure 1(a)), but in the sevoflurane group, the apoptosis caused by hypoxia was alleviated (Figure 1(b)). This confirmed that sevoflurane inhibited apoptosis.

The morphology of the cells did not change after hypoxia or sevoflurane treatment (Figure 2(a)).

In the same culture condition, the cell proliferation ability and cell density decreased after hypoxia treatment. The addition of sevoflurane alleviates the cell loss. In the cell survival assay, the cell survival index of hypoxia treatment was significantly lower than that of the control group (Figure 2(b)). Similar to the results of apoptosis test, the proliferation ability of cells treated with sevoflurane was enhanced.

To investigate the molecular biological causes of sevoflurane's inhibition of hypoxic cell apoptosis, western blot was used to detect protein expression. Apoptosis-promoting proteins such as CHOP, CRP78, and BAX were significantly increased in the hypoxia group, while apoptosis-inhibiting protein Bcl-2 was significantly higher in the sevoflurane group than in the hypoxia group (Figures 3(a) and 3(b)). This explains why the apoptosis of sevoflurane-treated cells was significantly lower than that of the hypoxia group.

In addition, we examined intercellular adhesion molecule-1 (ICAM-1), vascular cell adhesion molecule-1 (VCAM-1), and E-selectin proteins, which are thought to be expressed in the presence of myocardial injury. Western blot detection revealed that these proteins were highly expressed in 12-hour hypoxic cardiomyocytes and significantly decreased in cells treated with sevoflurane (Figures 4(a) and 4(b)). This revealed the protective effect of sevoflurane on myocardial cells during anesthesia.

## 4. Discussions

Commonly used inhalation drugs for volatile general anesthesia include halothane, isoflurane, sevoflurane, and other internal halogenated alkanes [12]. Pain, high price, and nonexplosive characteristics are widely favored by patients and doctors. With the increase in frequency and dosage, halothane anesthesia is gradually exposed to poisons in various systems of the body, in addition to degenerative damage to the nervous system, liver cancer damage, and cardiovascular suppression [13]. The anesthetic drug sevoflurane has the characteristics of rapid induction and depth of anesthesia, and many studies have shown that sevoflurane has a lighter cardiovascular inhibitory response and has a certain myocardial protective effect [14, 15].

Early structural and functional damage to vascular endothelial cells is the basis of the pathophysiology of I/R injury, and vascular endothelial cells are oxygen free radicals, adhesion molecules, and other biologically active substances during I/R injury source [16]. Autophagy plays an important role in the pathogenesis and progression of cardiovascular diseases such as myocardial ischemia-reperfusion, myocardial infarction, and heart failure. Excessive autophagosome accumulation and autophagy activation were observed in mouse undergoing myocardial I/R injury, thereby contributing to cardiomyocyte death [16]. Furthermore, autophagy is also thought to participate in ischemic postconditioning-mediated cardioprotection [16]. Nonetheless, the function of autophagy in this process is complicated considering it plays a promoting or suppressing role in cardioprotection.

Apoptosis is the programmed death of type I cells performed by activated caspase (Caspase), which is a highly evolved gene-regulated cell process, which eliminates cells without producing harmful substances [17, 18]. Apoptosis is involved in acute and chronic loss of cardiomyocytes in various cardiovascular diseases, such as myocardial infarction, ischemic heart disease, various cardiomyopathy, and heart failure, and inhibiting apoptosis is a potential way to treat cardiovascular disease.

Sevoflurane postconditioning (SpostC) has previously been shown to enhance cardiac resistance to I/R injury in experimental and clinical studies [10, 11]. SpostC was used to treat Sprague-Dawley rats with I/R injury, and the data showed that SpostC dramatically reduced the infarct size and improved cardiac function by activation of the ERK pathway [19]. SpostC promoted autophagosome clearance in vitro, reduced cell damage, and enhanced cell viability to reduce hypoxia-reoxygenation (H/R) injury in H9C2 cells. Another study showed that the SpostC-induced cardioprotection in I/R injury in Sprague-Dawley rats was modulated by the activation of the PI3K/Akt/mTOR pathway, and SpostC protected mitochondrial functions and had an antiapoptotic role in I/R-injured rats [20]. SpostC protects the heart from I/R injury through multiple mechanisms that involve the nuclear factor-erythroid-2-related factor-2 (NRF2) pathway, the reduction of reactive oxygen species (ROS) levels, and extracellular signal-regulated kinase (ERK) phosphorylation [21–24].

Oxidative stress and inflammation-induced endothelial dysfunction play a critical role in the pathogenesis of cardiovascular diseases. The anesthetic confers cytoprotective effects by virtue of its anti-inflammatory properties in various pathologies such as systemic inflammatory response syndrome and I/R injury. Sevoflurane, one of the most commonly used anesthetics, was proven to be effective in combating oxidative stress and inflammation and protecting organs against stress-induced injury in various conditions. Sevoflurane preconditioning could greatly attenuate tumor necrosis factor *α*- (TNF-*α*-) induced permeability and activation of p38 MAPK in rat pulmonary microvascular endothelial cells by reducing ICAM-1 expression. In our study, the expression of adhesion proteins in sevoflurane-treated myocardium was higher than that in myocardium treated with hypoxia, suggesting better connectivity of the myocardium.

Sevoflurane, as a commonly used anesthetic, has the characteristics of fast onset and easy regulation. Many studies have shown that sevoflurane inhibits cardiovascular responses less. Moreover, some evidence suggests that sevoflurane has a protective effect on the heart. It also affects the expression of various cytokines such as tumor necrosis factor (TNF-*α*), ICAM-1 in endothelial cells, and the level of cellular inflammation.

We used rats as model organisms and used in vitro cultured primary cells for hypoxia modeling. Our results revealed that sevoflurane treatment could reduce apoptosis of cardiomyocytes, similar to previous conclusion that sevoflurane ameliorated H/R-induced cardiomyocyte apoptosis by autophagy inhibition via reducing Beclin-1/PI3KC3 formation and PI3KC3 activity [25]. Also, our conclusion was consistent with Yu et al., who described that the cardiomyocyte apoptosis inhibited by sevoflurane postconditioning may influence the modulation of the expression of pro- and antiapoptotic proteins, specifically Bcl-2, BAX, and phosphor-Bad [26]. Besides, the study has indicated that sevoflurane could significantly improve the hypoxia-reoxygenation injury of the rats via decreasing the apoptosis of cardiomyocytes [27].

Collectively, our study provides evidence for the effect of sevoflurane on myocardial capacity and provides reference for clinical medicine. These preliminary findings require validation with further *in vitro* and *in vivo* studies. More studies should pay attention to investigating the roles of sevoflurane and the molecular basis for cardiac protection by sevoflurane *in vivo* (especially in human cardiac tissues) or in hypoxia injury in cardiomyocytes *in vitro*.

## Figures and Tables

**Figure 1:** The sevoflurane treatment group showed less apoptosis. (a, b) TUNEL staining demonstrated an increased apoptosis rate of myocardial cells in the hypoxia group. However, the apoptosis rate of myocardial cells in the hypoxia group was decreased after sevoflurane treatment. ^∗^*P* < 0.05 and ^∗∗^*P* < 0.01.

**Figure 2:** The survival ability of myocardial cells treated with sevoflurane increased compared with that treated with hypoxia. (a) The morphology of the cells did not change after hypoxia or sevoflurane treatment. (b) The cell viability test showed that the myocardial viability of the sevoflurane treatment group was significantly better than that of the hypoxia treatment group. ^∗^*P* < 0.05 and ^∗∗^*P* < 0.01.

**Figure 3:** Expression of apoptotic proteins in the hypoxia- and sevoflurane-treated groups. (a, b) Western blot was used to detect the expression of apoptotic proteins such as Bcl-2, CHOP, GRP78, and BAX. ^∗^*P* < 0.05 and ^∗∗^*P* < 0.01. ICAM-1: intercellular adhesion molecule-1; VCAM-1: vascular cell adhesion molecule-1.

**Figure 4:** Expression of cell adhesion protein in the hypoxia- and sevoflurane-treated groups. (a, b) Western blot was used to detect the expression of adhesion proteins such as ICAM-1, VCAM-I, and E-selectin. ^∗^*P* < 0.05 and ^∗∗^*P* < 0.01. ICAM-1: intercellular adhesion molecule-1; VCAM-1: vascular cell adhesion molecule-1.

## Data Availability

The authors confirm that the data supporting the findings of this study are available within the article.
